This article has been retracted.

# ML-Based Texture and Wavelet Features Extraction Technique to Predict Gastric Mesothelioma Cancer

**DOI:** 10.1155/2022/1012684

**Published:** 2022-07-04

**Authors:** Neeraj Garg, Divyanshu Sinha, Babita Yadav, Bhoomi Gupta, Sachin Gupta, Shahajan Miah

**Affiliations:** ^1^Department of Computer Science and Engineering, Maharaja Agrasen Institute of Technology, Delhi, India; ^2^Department of Computer Science, Sushant University, India; ^3^School of Engineering and Technology, MVN University, India; ^4^Department of Information Technology, Maharaja Agrasen Institute of Technology, Delhi, India; ^5^Department of EEE, Bangladesh University of Business and Technology (BUBT), Dhaka, Bangladesh

## Abstract

Microsatellites are small, repetitive sequences found all across the human genome. Microsatellite instability is the phenomenon of variations in the length of microsatellites induced by the insertion or deletion of repeat units in tumor tissue (MSI). MSI-type stomach malignancy has distinct genetic phenotypes and clinic pathological characteristics, and the stability of microsatellites influences whether or not patients with gastric mesothelioma react to immunotherapy. As a result, determining MSI status prior to surgery is critical for developing treatment options for individuals with gastric cancer. Traditional MSI detection approaches need immunological histochemistry and genetic analysis, which adds to the expense and makes it difficult to apply to every patient in clinical practice. In this study, to predict the MSI status of gastric cancer patients, researchers used image feature extraction technology and a machine learning algorithm to evaluate high-resolution histopathology pictures of patients. 279 cases of raw data were obtained from the TCGA database, 442 samples were obtained after preprocessing and upsampling, and 445 quantitative image features, including first-order statistics of impressions, texture features, and wavelet features, were extracted from the histopathological images of each sample. To filter the characteristics and provide a prediction label (risk score) for MSI status of gastric cancer, Lasso regression was utilized. The predictive label's classification performance was evaluated using a logistic classification model, which was then coupled with the clinical data of each patient to create a customized nomogram for MSI status prediction using multivariate analysis.

## 1. Introduction

Gastric cancer is one of the most common malignant tumors in the world. There were 1,033,701 new cancer cases, accounting for 5.7% of the global new cancer cases, and 782, 685 deaths, accounting for 8.2% of global cancer deaths. It ranks fifth in cancer incidence and third in mortality, and there is no decreasing trend in the incidence rate [1]. The heterogeneity of cancer, the appearance of gastric cancer, and the complex and diverse cancer types make the diagnosis and treatment of cancer more difficult. Microsatellite instability results from an impaired DNA mismatch repair, and a specific cancer phenotype is characterized by hypervariability of short repeats in the genome, a form characterized by DNA polymerase slippage and single nucleotides [2]. Extensive lengths of the microsatellite repeats are due to increased frequency of variants (SNVs). Polymorphism studies have shown that MSI-type gastric cancer accounts for about 15% of gastric cancer patients; these patients are more likely to benefit from immunotherapy [3]. MSI-type gastric cancer patients have their unique clinical features, such as the diffuse cancer tissue genome which is less stable, the disease site which is often distal to the tumor tissue, and the tumor types which are mostly type 3; MSI-type gastric cancer patients usually have a good overall long-term prognosis, compared with the contemporary MSS-type gastric cancer patients; for MSI-type gastric cancer, the survival rate of patients is high [4]. From precancer to onset, MSI gradually accumulates and increases, and therefore, MSI detection for early diagnosis and screening of gastric cancer is prolonged [5]. The prognosis of gastric cancer patients and the clinical decision-making of adjuvant gastric cancer treatment are of great significance. There are two main methods of MSI detection: immunohistochemistry (Immunohistochemistry, IHC) and polymerase chain reaction (PCR). IHC responds to MSI by detecting the expression of mismatch repair gene state; PCR is carried out through a specific single-nucleotide site gene tagging genetic analysis; however, both IHC and PCR testing methods need to be large-capacity tertiary medical center and require high economic and time cost; it is difficult to extend to every patient in clinical practice [6]. Therefore, none provides timely immune screening for a large number of potential immunotherapy-sensitive patients with point inhibitor therapy, thereby losing the chance to control the disease [7].

Histopathology is an essential tool for cancer diagnosis and prediction, and its type reflects the combined effects of molecular changes on cancer cell behavior. Assessing disease progression provides a direct visualization tool. A group of histopathologists can assess cell density, tissue structure, and histological filamentous features such as cleft status which were used to classify lesions. Along with advances in microscopy, imaging technology, and computer technology based on pathological pictures, auxiliary diagnostic models are developing rapidly. Among them, image texture analysis is used for pathology. Image texture feature extraction for cancer grading, Classification and predict for example, the author [8]. For extracting tissue disease from breast cancer patients, the grayscale co-occurrence matrix (GLCM) and the graph run-length matrix (GRLM) of the image is used. Euler number and other texture features, using Linear Discriminant Classifier (LDA) are used to map histological images, malignant and non-malignant histopathology Image, and the classification accuracy was 80% and 100%, respectively. The researcher in this study has done extracting three sets of texture features of soft tissue sarcoma: gray level cooccurrence matrix (GLCM), gray-level run-length matrix (GLRLM), and local binary modulus texture analysis using the LBP method to achieve the metastases and lesions of soft tissue sarcoma's death prediction [9]. Author has trained a deep convolutional neural network; two subtypes of lung cancer can be accurately distinguished from histopathological images: lung adenocarcinoma (LUAD) and lung squamous cell carcinoma (LUSC). Mutation status of six genes is associated with lung cancer. In this study, tumors, malignancy of the lymph node is a predictor that has consequences for the degree of lymph dissection. Numerous nodal units are engaged in the capillary permeability of the stomach, each with a variable risk of malignancy. This study aimed to construct a deep network system for predicting lymph cancer in numerous nodal sites in individuals with gastric cancer using preoperative CT data. ML techniques are employed for the examination of these CT scans for the investigation of any changes if occurred to predict the ailments and recommend precautions for better curability [10]. The focus of this research was to see if radiomic evaluation employing spectroscopic micro-CT-enhanced nanoparticle contrast enhancing may help distinguish tumors dependent on the amount of malignant cell lymphocytes [11]. In this research to improve survival prognosis, we offer a unique combined multitask system with multilayer characteristics that predicts clinical tumor and metastasis stages simultaneously to detect gastric cancer [12]. This paper can establish to fuse the statistical model of multiple residual networks; it can be obtained from a standard hematoxylin and accurate prediction of prostate cancer patients in histopathological images after eosin staining the mutation status of the speckle-type POZ gene [13].

This paper proposes gastric cancer based on the texture features of histopathological images. Authors in this research have forecasted MSI prediction method that targets tumor heterogeneity in gastric cancer histopathology, where researchers have used image feature extraction technology and a machine learning algorithm to evaluate high-resolution histopathology pictures of the patients. 279 cases of raw data were obtained from the TCGA database, out of which 442 samples were acquired after preprocessing and upsampling, and 445 quantitative image features, including first-order statistics of impressions, texture features, and wavelet features, were extracted from the histopathological images of each sample. To filter the characteristics and provide a prediction label (risk score) for MSI status of gastric cancer, Lasso regression was employed. Furthermore, the predictive label's classification performance was evaluated using a logistic classification model, which was then coupled with the clinical data of each patient to create a customized nomogram for MSI status prediction using multivariate analysis as an achievement of the research.

### 1.1. Organization

The paper is outlined in several sections where the starting section is the introduction part followed by the second section which discusses the data and methods employed in the study. The third section defines the analysis of experimental results, followed by the penultimate section that states about discussions and findings, and the ultimate section is the conclusion of the study.

In the representation of Figure 1 as depicted below, the extracted quantitative image features from images have been acquired, and the use of Lasso regression to construct the prediction has targeted a signature, and using the predictive signature as an independent predictor to be combined with the patient's clinical features has been opted, additionally the multivariate analysis by logistic regression to build a predictive model has been obtained; at last the prediction tool is being drawn termed as nomogram of personality that provides a powerful instrument for MSI prediction in gastric cancer patients. The method of flow is shown in the figure below.

## 2. Data and Methods

### 2.1. Patient Data

This paper's histopathological images of gastric cancer are from the TCGA data library. In addition, the MSI status of gastric cancer patients was analyzed to use the obtained data effectively. This study established three inclusion criteria for the collected data: (1) Pathological images showing uniform staining, precise imaging and no tissue adhesion; (2) uniformly complete personal basic information and clinical characteristics; (3) have clear MSI status information. After screening, 277 case samples were eligible for the inclusion standard.

### 2.2. Data Preprocessing

To ensure the validity of the experiment and obtain valuable results, it is necessary to solve the problem of sample imbalance. Augment the minority class by sampling. For MSI-type cases, histopathological images for each patient is considered. Select multiple ROIs, each ROI as an independent sample, upsampled. The dataset has a total of 442 pieces. The obtained models are randomly divided into a training set and a validation set: There are 313 samples in the training set, of which 156 are of MSI type. There are 157 cases of MSS type; there are 129 samples in the validation set, of which 64 cases are of MSI type, for example, 65 cases of MSS type.

### 2.3. Image Segmentation

The histopathological image needs to be processed before image feature extraction to ensure the accuracy of the resulting image features and reduce the computational complexity degree segmentation. To obtain the most representative lesion area, under the guidance of a chief physician with experience in histopathological image detection, the tumor area was annotated and examined the marked lesion area by another expert. Finally, the ROI of all histopathological images was obtained by segmentation.

### 2.4. Feature Extraction

In this study, the original image of the ROI is obtained from the segmentation and the processed wavelet. A total of 445 image features are extracted from the filtered image, which can be divided into two classes, six groups per class: first-order statistics and gray-level cooccurrence matrix (GLCM), gray-level size zone matrix (GLSZM), gray-level run-length matrix (GLRLM), neighboring gray tone difference matrix (NGTDM), and gray-level dependence matrix (GLDM).

First-order statistics describe interest through common statistical indicators pixel intensity distribution within the region of interest. GLCM describes the grayscale of an image and the second-order joint probability function of the spatial correlation characteristics obtained by calculating GLCM using the partial eigenvalues of the matrix to represent the texture features of the image, which can give the comprehensive information about the direction, adjacent interval and changing amplitude of the grayscale of the response image [14]. GLSZM is used to quantify the gray-level area in the image; the gray-level area domain is defined as the number of connected pixels that share the same gray-level intensity. GLRLM is used to quantify grayscale runs, which are defined as the length of consecutive pixels of the same gray value. In NGTDM through grayscale, the sum of absolute differences reflects the difference between the average gray values of adjacent pixels different. GLDM can quantify the grayscale dependence in images; grayscale dependence is defined as the number of connected pixels within a distance *δ* that depends on the center pixel [15].

This study extracted 18 features from first-order statistics, mainly including entropy, total energy, mean absolute deviation, and skewness; from GLCM, 22 kinds of features are extracted, mainly including autocorrelation, joint average, clustering shading, and cluster tendency; 16 features were extracted from GLSZM, mainly including grayscale uneven normalization, uneven area size, and area percentage size area nonuniformity normalization; 16 were extracted from GLRLM features, including run entropy, run difference, gray variance, and run nonuniformity uniform standardization; 5 kinds of features are extracted from NGTDM, mainly including roughness, contrast, complexity, and intensity; 14 were extracted from GLDM features, mainly including dependence entropy, dependence nonuniformity, dependence nonuniformity standard standardization, and dependent variance.

### 2.5. Feature Selection

To reduce the complexity of the model and prevent overfitting, before modeling, this paper, features are selected using the lasso method [16]. Lasso improves the traditional, linear regression method provides a new perspective on the general linear regression algorithm on the basis of adding the L1 penalty term, the linear regression parameters have sparsity from the resulting model which has good predictability, and the selected features are related to the prediction. The test label is more relevant. For the feature vector *xi* (*i* = 1, 2, ⋯, *N*) of a given sample, *xi* ∈ *Rn*. The objective function of Lasso regression is

(1) $$\begin{array}{c} L\left(\alpha ,\gamma \right)=\overset{N}{\underset{i=1}{\sum }}{\left(y_{i}-\underset{j}{\sum }x_{ij}a_{j}\right)}^{2}+\gamma \overset{p}{\underset{j=1}{\sum }}\left|a_{j}\right|, \end{array}$$

where *y* is the label of the sample and *α* = {*aj*} is the regression parameter to get the most optimal regression parameters and transform the objective function minimization problem into the following subproblems:

(2) $$\begin{array}{c} a_{j}^{\left(k+1\right)}=\text{argmin}\frac{L}{2}{\left\|a-z_{j}\right\|}_{2}^{2}+\gamma {\left\|a\right\|}_{1} \end{array}$$

In:

(3) $$\begin{array}{c} z_{j}=a_{j}^{\left(k\right)}-\frac{1}{L}\nabla f\left(a_{j}^{\left(k\right)}\right), \end{array}$$

(4) $$\begin{array}{c} \nabla f\left(a_{j}^{\left(k\right)}\right)=2\overset{N}{\underset{i=1}{\sum }}\left[x_{ij}\left(\overset{P}{\underset{s=1}{\sum }}x_{\text{is}}a_{s}^{\left(k\right)}-y_{i}\right)\right]. \end{array}$$

Using proximal gradient descent [17], the algorithm iteratively solves Equation (3) and uses the soft domain function to solve Equation (2); the final solution is as follows:

(5) $$\begin{array}{c} a_{j}^{\left(k+1\right)}=\left\{\begin{array}{c} z_{j-\left(\gamma /L\right),z_{j}>\left(\gamma /L\right),}\\ 0,\left|z_{j}\right|\leq \frac{\gamma }{L},\\ z_{j}+\frac{\gamma }{L},z_{j}<\frac{\gamma }{L}. \end{array}\right. \end{array}$$

Through the above algorithm, the sparse feature matrix is finally obtained, which is used to build a classification model.

### 2.6. Predictive Label Construction

In this study, the sparse eigenvalues and their regression coefficients were used to construct a sample.  Table 1 shows the risk score of the proposed model over the number of features and log variance. In the predicted label of Ben, the formula is as follows:

(6) $$\begin{array}{c} \text{Risk score}=\overset{n}{\underset{i=1}{\sum }}{Feature}_{i}\times \alpha_{i}. \end{array}$$

Among them, feature is the *i*^th^ eigenvalue of the sample feature vector, and *α*_*i*_ is the regression coefficient corresponding to the eigenvalue.  Table 2 shows the risk coefficient of the proposed model over the number of feature and log variance.

Using risk score as an independent predictor and the clinical samples, combine features to build logistic regression models and draw personalized nomogram picture and through C index, AUC value, calibration curve, and decision curve evaluation predictive performance of the model [18].

## 3. Analysis of Experimental Results

### 3.1. Clinical Features

The histopathological images used in this study were obtained from 277 gastric cancer patients, including 55 patients with MSI-type gastric cancer and 222 patients with MSS-type gastric cancer. Among them, there were 188 male patients and 89 female patients, with a median age of 67.64 years (33-90 years old), and the prevalence of MSI was 19.85% (55/277). According to gastric cancer, patients were divided into two groups by MSI status. There are differences in gender, age, and TNM staging between patients and MSS patients. The clinical characteristics of the patients are shown in Table 3.

### 3.2. Image Feature Screening and Predicted Label Construction

Based on the MSI status, Lasso regression is applied on the training set, features are filtered, and Figure 2(a) shows the binomial error classification points with log *γ*, where the least binomial error classification point represents the most retained. The best number of features fit the model. Based on the minimum criterion and 1 standard error standard, with 10-fold cross-validation, draw the dashed vertical with the best *γ* value wire.  Figure 3(b) shows the lasso coefficient curve of the image features [19].

The results of lasso regression are shown in Tables 4, and 9 lines were finally screened nonzero number of features, including 4 image features based on the original image and based on 5 image features after wavelet filtering. Calculate the sample by Formula (6) Ben's risk score. Single-factorial correlation of 9 image features with MSI status and prime variance analysis shows that the *P* values were all less than 0.001, indicating that the characteristics obtained from the screening were closely related to gastric MSI status of cancer patients and was significantly correlated.

### 3.3. Prediction Accuracy Verification

Based on the selected image texture features and logistic regression training, a predictive classification model for MSI was constructed. As shown in Figure 3, the ROC curve in line analysis, the AUC value was 0.75. Then apply that model to the validation set which can effectively predict MSI status in ROC curve analysis, AUC. The value is 0.74. Therefore, 9 features constituting the model associated with gastric cancer histopathological image features associated with patients' MSI status.  Table 5 gives the results of each evaluation index of the classification model [20].

### 3.4. Construction and Evaluation of Monogram

To reflect the clinical value of the predictive model, this study used all datasets.  Table 6 and Figure 4 show the model evaluation results.

The Nomo-gram based on clinical characteristics were constructed using Risk Score. The latter nomogram was used to predict the MSI status of gastric cancer patients, as shown in Tables 7 and 8.

The nomogram includes gender, age, TNM stage, and risk score, which allows users to obtain MSI status predictions corresponding to patient covariate combination probability. For example, locate the patient's TNM stage axis; draw a line on that axis a vertical line to determine the predicted score corresponding to that TNM stage. For each variable, repeat this process and add the scores for each covariate to make the total score corresponding to get the predicted probability to achieve the MSI status of gastric cancer patients predict.

Apply the index of concordance (C-index), respectively, AUC, and calibration curve to evaluate the predictive performance of the nomogram. AUC values before and after adding risk score were 0.696 and 0.802; the consistency index is shown in Table 9; after adding risk score, the value of C-index is improved from 0.69. The calibration curve is shown in Figure 5. The dotted line represents the ideal prediction state. The results show that the calibration curve fits better after adding the prediction label constructed in this study.  Table 10 shows the Calibration Curve Comparisons.

To further validate the clinical utility of the predictive model, a decision curve line analysis to quantify the net gain to evaluate columns based on texture features of pathological images was done. As shown in Figure 6, in the entire risk threshold area during the period, the predictive model after adding risk score achieved a larger net income beneficial.  Table 11 shows the decision curve comparison.

This result shows that adding the risk score nomogram has a greater bed application potential.

### 3.5. Comparison with Other MSI Prediction Studies

To further verify the performance of the model, other studies on MSI prediction were compared, and the comparison results shown in Table 12 developed three prediction models for MSI prediction by extracting the morphology, texture, Gabor wavelet, and other radiomic features of CT images, combined with clinical features, using Lasso and Naive Bayes classifiers, and using clinical features alone [21]. The AUC value of the model with radiomic features was 0.598, the AUC value of the model using radiomic features alone was 0.688, and the AUC value of the model combining radiomic and clinical features was 0.752, which has a large gap with the classification performance of the proposed MSI prediction model.

Win trained a ResNet-18 network through the slices of histopathological images to obtain the likelihood distribution of the patient's MSI status, generated the plaque likelihood histogram feature, and used the XGBoost classifier to predict the patient's MSI status [22]. The model has an AUC value of 0.93 on the training set and 0.73 on the test set, indicating obvious overfitting.

## 4. Discussion and Findings

This paper proposes a texture feature based on histopathological images of gastric cancer. The MSI prediction method of sign was used to extract the texture features such as GLCM, GLSZM, GLSZM, and GLRLM. In these texture features, after wavelet transformation sign, we have employed Lasso regression for feature selection, and lastly the texture features most relevant to the MSI state of the user are constructed based on these texture features. The MSI prediction labels of gastric cancer were obtained, and the predictions were compared on the training and validation sets. The label classification performance is verified, and the AUC values obtained are 0.75 and 0.74, respectively. The results show that the proposed predictive signature has a better effect on the MSI status of gastric cancer patients compared with the traditional MSI detection methods initially opted, using machine learning technology based on direct prediction of MSI in gastric cancer patients on the basis of readily available histopathological image status, without the need for additional laboratories for genetic testing and immunohistochemistry analysis; the prediction of MSI status can be achieved at a lower cost. Hence, this method when compared to computer-aided MSI prediction methods based on CT images outperforms, because the reproducibility of radiology features considering different scanners and imaging protocols and the potential differences in terms of the formation of H&E-stained histopathological images are less stable comparing to the performance of the MSI prediction model proposed in this paper. Therefore, this investigation proposes and confirms a strategy for predicting MSI in gastric cancer based on histopathological pictures that may accurately predict the MSI status of patients with gastric cancer, allowing for universal MSI screening and benefiting more gastric cancer patients to be investigated in a significant manner.

## 5. Conclusion

This study proposes and validates a method for predicting MSI in gastric cancer based on histopathological images, which can effectively predict the MSI status of patients with gastric cancer, hence providing a possibility for universal screening of MSI, and is expected to benefit more gastric cancer patients. Immunotherapy by combining the clinical features with predictive labels is proposed in this paper to construct gastric cancer MSI prediction models, as compared with prediction models based on clinical characteristics; after entering the predicted labels that are proposed in this paper, the AUC value of the model is improved from 0.696 to 0.802. To further verify the validity of the predicted labels, the clinical value of sex and predictive models, respectively, before and after adding predictive labels are analyzed. The prediction model was evaluated by calibration curves, C-index values, and decision curves. The results show that after adding the predicted labels proposed in this paper, the C-index value and the calibration performance of the quasi-curve are significantly improved, and the decision curve analysis has also demonstrated a greater net income.

## Figures and Tables

**Figure 1:** Construction process of MSI prediction model for gastric cancer.

**Figure 2:** Lasso regression process.

**Figure 3:** ROC curves of training set and test set.

**Figure 4:** Model evaluation results.

**Figure 5:** Calibration curve comparisons.

**Figure 6:** Decision curve comparison.

**Table 1:** Risk score of the proposed model over the number of features and log variance.

Log *γ*	Binomial deviance	Number of features
-2	1.4	2
-4	1.35	5
-6	1.3	5
-8	1.25	9
-10	1.2	12

**Table 2:** Risk coefficient of the proposed model over number of feature and log variance.

Log *γ*	Coefficients	Number of features
-2	10	12
-4	5	11
-6	3	8
-8	2.5	11
-10	5	12

**Table 3:** Clinical characteristics of the patients.

Feature item	Classification	MSI (*n* = 55)	MSS (*n* = 222)	*P* value
Age	Mean	70.91	63.74	<0.001∗∗∗
	Range	46~90	36~90	
Gender	Male	35 (54.5%)	157 (71.2%)	<0.001∗∗∗
	Female	25 (45.5%)	64 (28.8%)	
TNM stage	I	12 (21.8%)	25 (11.3%)	<0.001∗∗∗
	II	20 (36.4%)	67 (30.1%)	
	III	19 (34.5%)	106 (47.7%)	
	IV	4 (7.3%)	24 (10.8%)	

**Table 4:** Lasso regression results.

Feature name	Regression coefficients	*P* value
original_firstorder_10Percentile	0.212 204	<0.001∗∗∗
original_firstorder_90Percentile	0.404 922	<0.001∗∗∗
original_firstorder_Median	6.118 815	<0.001∗∗∗
original_firstorder_Skewness wavelet-	-0.817 240	<0.001∗∗∗
HL_glcm_Imc2 wavelet-	-0.650 800	<0.001∗∗∗
LL_firstorder_10Percentile wavelet-	0.490 395	<0.001∗∗∗
LL_firstorder_Median wavelet-	-5.750 580	<0.001∗∗∗
LL_glcm_ClusterShade wavelet-	1.133 542	<0.001∗∗∗
LL_glrlm_GrayLevelEmphasis	-0.254 150	<0.001∗∗∗

**Table 5:** Each evaluation index of the classification model.

Log *γ*	True positive rate	False positive rate	Train Auc:0.74	Train Auc:0.75
-2	0	0	0.1	0.1
-4	0.2	0.2	0.16	0.18
-6	0.45	0.45	0.21	0.25
-8	0.65	0.65	0.45	0.48
-10	0.85	0.85	0.71	0.75

**Table 6:** Model evaluation results.

Dataset	Precision	Recall	F1 value	AUC value
Training set	0.68	0.73	0.72	0.75
Validation set	0.65	0.67	0.67	0.74

**Table 7:** Evaluation results of model (before joining risk score).

Points	0-100
Gender	0 or 1
Age	30-90
TNM stage	01-Apr
Total point	0-180
Linear predictor	[-2.5,2.5]
Risk of MSI	0.1-0.9

**Table 8:** Evaluation results of model (after adding risk score).

Points	0-100
Gender	0 or 1
Age	30-90
TNM stage	01-Apr
Risk score	[-3.5,3.0]
Total point	0-130
Linear predictor	[-4,3]
Risk of MSI	0.1-0.9

**Table 9:** C-index evaluation of prediction model.

Predictive model	C-index	95% CI
Before joining risk score	0.7	0.64~0.74
After joining risk score	0.8	0.76~0.84

**Table:** (a) Before joining risk score

Actual probability	Predicted probability	Apparent	Bias-corrected	Ideal
0	0	0	0	0
0.2	0.2	0.1	0.09	0.2
0.4	0.4	0.43	0.42	0.4
0.6	0.6	0.58	0.55	0.6
0.8	0.8	0.78	0.75	0.8

**Table:** (b) After joining risk score

Actual probability	Predicted probability	Apparent	Bias-corrected	Ideal
0	0	0	0	0
0.2	0.2	0.2	0.19	0.2
0.4	0.4	0.38	0.35	0.4
0.6	0.6	0.7	0.68	0.6
0.8	0.8	0.79	0.78	0.8

**Table 11:** Decision curve comparison.

Net benefit	High-risk threshold	Clinical feature	Risk score + clinical feature	ALL
-0.05	0	0.3	0.3	0.3
0	0	0.26	0.28	0.3
0.05	0.2	0.2	0.25	0.15
0.1	0.4	0.16	0.19	0
0.15	0.6	0.1	0.15	0
0.2	0.8	-0.01	-0.01	0
0.25	0.9	0.03	0.1	0
0.3	1	0	0	0

**Table 12:** Performance comparison of MSI prediction models.

Method	Type of data	Image features	Clinical features	Joint model
Win	Histopathological images	0.74	_____	______
Nano	CT image	0.68	0.599	0.755
Proposed model	Histopathological images	0.75	0.697	0.801

## Data Availability

The data shall be made available on request.
